# Microplasma Synthesis of Antibacterial Active Silver Nanoparticles in Sodium Polyacrylate Solutions

**DOI:** 10.1155/2021/4465363

**Published:** 2021-10-19

**Authors:** Mariana Shepida, Orest Kuntyi, Yuriy Sukhatskiy, Artur Mazur, Martyn Sozanskyi

**Affiliations:** Lviv Polytechnic National University, Lviv 79013, Ukraine

## Abstract

The great demand for functional, particularly biologically active, metal nanoparticles has led to the search for technologically effective, green, and controlled methods of synthesizing these metal nanoparticles. Plasma glow discharge is one of the most promising techniques in this direction. The results of studies based on the synthesis of colloidal solutions of stabilized silver nanoparticles (AgNPs) by the microplasma method in solutions of a nontoxic surfactant sodium polyacrylate (NaPA) are presented. It is shown that AgNPs with a size of 2–20 nm are formed in solutions of 0.05–0.2 mmol·L^−1^ AgNO_3_ + 5 g·L^−1^ NaPA at *U* = 250 V by tungsten cathode plasma glow discharge. At 20°C, the yellow solutions are formed with *λ*_max_ ≈ 410 nm, which are stable during long-term storage. It was found that the process of AgNPs formation corresponds to a first-order reaction on the AgNO_3_ concentration. Its value has little effect on the geometry of nanoparticles, so the Ag(I) concentration in solution is one of the main factors influencing the rate of microplasma synthesis of AgNPs. The antimicrobial activity of synthesized AgNPs solutions against strains of *Escherichia coli*, *Staphylococcus aureus*, and *Candida albicans* was established.

## 1. Introduction

Metal nanoparticles, especially silver nanoparticles, demonstrate high efficiency in medicine [1–3], sensing [4], catalysis [5], and the agrifood sector [6]. Considering the dependence of the functional properties of MNPs on their shape and size, and in the case of M_1_M_2_NPs, also dependent on the content of components, significant attention has been paid in the last decade to synthesis methods. After all, they are decisive in forming the structure (composition) of nanoparticles and, accordingly, their properties. Therefore, the controlled synthesis of nanoparticles is one of the main criteria in choosing a method. The defining criteria also include engineering and “green” technology. The latter is the most studied for the use of these three major biological sources: plant extract [5, 7], bacteria [2, 3, 6, 8], and fungi [9]. All of them contain components, which are necessary for the synthesis of colloidal solutions of stabilized metal nanoparticles with the help of reductants, which reduce metal ions (1) and surfactants, which after the formation of MNCs and MNPs (2), provide their stabilization (3).

(1) $$\begin{array}{c} {\text{M}}^{\text{n}+}+\text{ ne}\left(\text{biol.reduc.}\right)⟶{\text{M}}^{\text{0}} \end{array}$$

(2) $$\begin{array}{c} {\text{mM}}^{\text{0}}⟶{\text{M}}_{m}^{0} \end{array}$$

(3) $$\begin{array}{c} {\text{M}}_{m}^{0}+\text{ biol.surf.}⟶\text{Agn@biol.surf.} \end{array}$$

Sonochemical and sonoelectrochemical production of nanoparticles [10] and plasma glow discharge [11–13] are effective for increasing the rate of processes similar to (1)–(3). Plasma electrolysis is one of the relatively new and promising methods for the synthesis of nanomaterials. Significant attention is paid to the microplasma, which is characterized by a relatively low temperature and, at the same time, high “density” of electrons. This is especially important for synthesizing colloidal solutions of metal nanoparticles using surfactants. Plasma electrolysis allows the controlled formation of particle geometry, which is one of the main requirements of modern nanotechnology. It is also worth noting that plasma meets the requirements of green technologies. This is because plasma does not provide for the use of reducing reagents

A feature of the microplasma is the generation of electrons (е^−^) during the discharge, which are hydrated in aqueous solutions (4). The latter (е^−^_aq_) reduce metal ions (5) and cause the formation of H· and OH radicals and new compounds, in particular, H_2_O_2_ [14]. Some of them are reducing agents for many metal ions (6) and (7). Microplasma synthesis is characterized by its high rate and the absence of a chemical reductant, which minimizes the number of precursors. This method allows using surfactants as stabilizers of MNCs and MNPs, which allows a controlled influence on the formation of their geometry during the stages of nucleation and growth (8).

(4) $$\begin{array}{c} {\text{e}}^{-}+{\text{H}}_{2}\text{O}⟶{\text{e}}_{\text{aq}}^{-} \end{array}$$

(5) $$\begin{array}{c} {\text{M}}^{\text{n}+}+{\text{ne}}_{\text{aq}}^{-}⟶{\text{M}}^{\text{0}} \end{array}$$

(6) $$\begin{array}{c} {\text{M}}^{\text{n}+}+\text{ nH}\cdot ⟶{\text{M}}^{\text{0}}{+\text{ nH}}^{+} \end{array}$$

(7) $$\begin{array}{c} {\text{M}}^{\text{n}+}+{\text{nH}}_{2}{\text{O}}_{2}⟶{\text{M}}^{\text{0}}+{\text{nH}}_{2}\text{O}+{\text{n/}2\text{O}}_{2} \end{array}$$

(8) $$\begin{array}{c} {\text{mM}}^{\text{0}}+\text{surf.}⟶\text{Mm }\left(\text{MNCs@surf.}\right)⟶\ldots ⟶\text{MNPs@surf.} \end{array}$$

The microplasma glow discharge method is used to synthesize mainly noble metal nanoparticles [14–30]. Studies in recent years indicate the possibility of obtaining nanoparticles from nonferrous metals [31–35]. The microplasma method is efficient for the synthesis of bimetal nanoparticles [36–44]. The synthesis of MNPs is often carried out in solutions containing surfactants or stabilizers (Table 1) that are nontoxic or of natural origin.

Surfactants are one of the main factors influencing the formation of MNCs and MNPs, as well as their functional properties and stability during long-term storage [33, 45–52]. The aim of the work is to study the regularities of microplasma synthesis of silver nanoparticles in sodium polyacrylate solutions and establish the conditions of their stable formation. Polyacrylate is a nontoxic synthetic polymeric anionic surfactant that is known to be an effective stabilizer for MNPs [50–56].

## 2. Experimental

Plasma synthesis of colloidal solutions of silver nanoparticles was performed in a thermostated reactor (Figure 1) with a volume of 100 ml under continuous agitation at 20°C. The platinum plate was used as an anode and tungsten (99.9% purity) wire (∅ = 0.1 mm with a working length of 5 mm) as a cathode. The following electrolytes were used for research: 0.05–0.2 mmol·L^−1^ AgNO_3_ and 5 g·L^−1^ NaPА (pH8). The acidity value of the solutions was adjusted with a 1 mol·L^−1^ solution of CH_3_COONa.

The synthesis was performed at *U* = constant = 250 V. The values of current and voltage over time during the glow discharge were measured with a recorder (MTech ADC-UI18), as shown in Figure 2.

TEM images were obtained using a transmission electron microscope JEM-I230 (JEOL, Tokyo, Japan) with an acceleration voltage of 80 kV. The samples for TEM investigations were prepared by drying 0.05 *μ*L of silver sol on the carbon grid at room temperature. The diameters of obtained AgNPs were determined using TEM images by comparing individual particle sizes with the scales presented on images. Theoretical calculations and processing of experimental data were carried out using the software Inconico Screen Calipers 4.0 and OriginPro 8.0. The statistical histograms were obtained using the Origin software pack with standard deviation values as nanoparticle size. In addition, NP size and density were determined by using the public domain Java image processing program ImageJ2.

The antibacterial activity of AgNPs was evaluated against Gram-negative *Escherichia coli* (*E. coli*) and Gram-positive bacteria *Staphylococcus aureus* (*S. aureus*) and *Candida albicans* (*C. albicans*). To do this, the bacteria were inoculated into Petri dishes with a solid selective nutrient medium for each species of microorganisms: yellow-salt agar for the culture of *S. aureus*, Endo agar for the culture of *E. coli*, and Sabouraud Agar for *Candida albicans.* Inoculation was performed after 1, 6, 18, and 48 hours of contact of bacteria with 0.8 mm solution of AgNPs. All the biological material was incubated at 310 K for 24 hours in a bacteriological incubator. Antibacterial activity was indexed by counting the number of microorganisms (CFU/mL).

## 3. Results and Discussion

At pH >6, the structural elements in the polymer chain of polyacrylate transform from the form of (–CH_2_–CH–COOН)_n_ into the anionic form of (–CH_2_–CH–COO^−^)_n_. The fraction of the anionic form increases with an increase in the concentration of ОН^−^ ions [52]. In sodium polyacrylate solutions, Ag^+^ cations form soluble [Ag_m_PА]^(n-m)-^ complexes [50, 51, 53]. The latter are transformed into stabilized nanoclusters and nanoparticles (9) during microplasma glow discharge due to the reduction of Ag (I) to Ag (0) by hydrated electrons and generated radicals and compounds. Stabilization occurs due to the formation of surface complexes between the [−СОО^−^] polymer chain of polyacrylate and silver atoms of AgNCs and AgNPs with the formation of a continuous protective layer of polymer surfactant [52].

(9) $$\begin{array}{c} {\left[{\text{Ag}}_{\text{m}}\text{PA}\right]}^{\left(\text{n}-\text{m}\right)-}+\left({\text{me}}_{\text{aq}}^{-}\text{,mH}\cdot {\text{,mH}}_{2}{\text{O}}_{2}\right)⟶{\left[\text{Ag}{\left(\text{0}\right)}_{\text{m}}\text{PA}\right]}^{\text{n}-}\left(\text{AgNCs@PA,AgNPs@PA}\right). \end{array}$$

During microplasma glow discharge, yellow solutions are formed with an absorption maximum of ∼410 nm, the value of which practically does not change during synthesis and long-term storage (Figure 3).

The UV-Vis spectra do not show intermediate absorption bands at 310 and 345 nm belonging to “magic” silver clusters of special stability [55, 56]. Their formation is characteristic during the reduction of Ag(I) in NaPA solutions, and they are converted into nanoparticles with the formation of “blue silver” that is characterized by wide absorption bands at 490–530 nm [54–56]. This difference can be explained by the features of glow discharge synthesis, which causes a high concentration of active reducing agents (mе^−^_aq_, mН·, and mH_2_O_2_) in the solution volume and, accordingly, a high rate of Ag(I) reduction process and the formation of AgNCs and AgNPs (9). Under such conditions, the stability of the “magic” silver clusters, which are charged and contain a small number of Ag atoms (Ag_8_^2+^, Ag_9_^+^) [57], is complicated.

The nature of the UV-Vis spectra with the absorption maximum of ∼410 nm does not change in a wide concentration range of AgNO_3_ (Figures 4(a)–4(c)).

Increasing concentration of AgNO_3_ increases the increment of optical density value at *λ*_max_ = 410 nm over time (Figure 5), which is identical to an increase in the formation rate of AgNPs (Figure 6).

Analysis of the obtained kinetic curves showed that the formation process of AgNPs during microplasma synthesis in the AgNO_3_−NaPA solutions corresponds to the following first-order reaction:

(10) $$\begin{array}{c} -\frac{d\left[{\text{Ag}}^{+}\right]}{dt}=k\cdot \left[{\text{Ag}}^{+}\right]\text{,}\\ \ln\left(\left[{\text{Ag}}^{+}\right]\right)=\ln\left({\left[{\text{Ag}}^{+}\right]}_{\text{0}}\right)-k\cdot t. \end{array}$$

The values of the rate constants of AgNPs formation process (*k*_*G*_) at initial AgNO_3_ concentrations of 0.05, 0.10, and 0.20 mol L^−1^ are close to – 0.212, 0.207, and 0.193 min^−1^, respectively.

The sizes of nanoparticles do not exceed 30 nm (Figure 7) and depend little on the concentration of Ag(I) ions. So, the latter can be considered one of the main factors influencing the rate of microplasma synthesis of stabilized silver nanoparticles.

As already mentioned, the value of the absorption maximum (∼410 nm) of the synthesized AgNPs solutions practically does not change during long-term storage (Figures 7(a) and 7(c) and 8).

All this indicates the stability of the geometry of the synthesized nanoparticles during long-term storage.

## 4. Antibacterial Activity of Synthesized AgNPs

The results of studies on the antibacterial properties of microplasma-synthesized AgNPs indicate their activity against Gram-positive bacteria *Staphylococcus aureus* ATCC No. 25923, Gram-negative bacteria *Escherichia coli* ATCC No. 25922 (Tables 2 and 3), and fungicidal bacteria *Candida albicans* ATCC No. 885–653 (Tables 4 and 5).

The *Staphylococcus aureus* ATCC 25923 strain is more resistant than the *Escherichia coli* ATCC 25922 and *Candida albicans* ATCC 885–653 strains. Thus, the bactericidal action of the synthesized colloidal AgNPs solutions against *Staphylococcus aureus* ATCC 25923 in the studied range of contact time (1–48 h) is manifested only when the concentration of the AgNO_3_ solution increases from 0.1 to 0.2 mmol L^−1^ (Tables 2 and 3 and Figure 9). Two different mechanisms can cause antibacterial and fungicidal properties of the synthesized AgNPs solutions: (1) fixation of silver nanoparticles on cell membranes and their penetration into the cell, followed by damage to the membrane and release of the cell contents; (2) release of Ag^+^ ions, which have bactericidal and fungicidal properties [58, 59]. The authors [60] consider that silver nanoparticles have the maximum antimicrobial action with a size of less than 10 nm, as shown in Figure 8(b), and 58% of the silver nanoparticles obtained by microplasma synthesis have sizes less than 10 nm.

## 5. Conclusions

In solutions of the nontoxic surfactant sodium polyacrylate (NaPA) and AgNO_3_ by tungsten cathode plasma glow discharge at 250 V, the stabilized silver nanoparticles are formed. At the precursor's concentration of 0.05–0.2 mmol·L^−1^ AgNO_3_ + 5 g·L^−1^ NaPA, AgNPs are formed with a size of 2–20 nm. At 20°C, the yellow solutions are formed with *λ*_max_ ≈ 410 nm, which are stable during long-term storage. The process of AgNP formation corresponds to a first-order reaction in the AgNO_3_ concentration. The latter value has little effect on the geometry of nanoparticles, so the Ag(I) concentration in solution is one of the main factors influencing the rate of microplasma synthesis of AgNPs. The antimicrobial activity of synthesized AgNPs solutions against strains of *Escherichia coli*, *Staphylococcus aureus,* and *Candida albicans* was established.

## Figures and Tables

**Figure 1:** Scheme of the device for plasma synthesis of silver nanoparticles.

**Figure 2:** Changing of values of current and voltage over time during glow discharge in NaPA solution.

**Figure 3:** The UV-Vis spectra of AgNPs at different time points of synthesis by microplasma discharge in 0.1 mmol·L^−1^ AgNO_3_ + NaPA (5 g L^−1^) solution, *t* = 20°C.

**Figure 4:** The UV-Vis spectra of AgNPs at different synthesis durations by microplasma discharge in 0.05 mmol L^−1^ (a), 0.1 mmol L^−1^ (b), and 0.2 mmol L^−1^ (c) AgNO_3_ in 5 g·L^−1^ NaPA solution, *t* = 20°C.

**Figure 5:** Dependences of the optical density of solutions at *λ*_max_ = 410 nm on synthesis duration.

**Figure 6:** Kinetic curves of AgNP growth (a) and dependences of AgNP growth rate (W_G_) on synthesis duration (b) at different concentrations of AgNO_3._

**Figure 7:** TEM images (a, c) and the size distribution histograms (b, d) of AgNPs, synthesized in 0.1 mmol·L^−1^ AgNO_3_ (a, b) + 5 g·L^−1^ NaPA solution and 0.2 mmol·L^−1^ AgNO3 (c, d) + 5 g·L^−1^ NaPA solution, *t* = 20°C.

**Figure 8:** (a) TEM images of AgNPs after 1 month and (b) the size distribution histograms.

**Figure 9:** Agar plate assays to assess the antibacterial activity of AgNPs with different concentrations (mmol·L^−1^) of AgNPs and different contact time durations.

**Table 1:** Conditions of microplasma synthesis of MNPs and M_1_M_2_NPs in aqueous solutions and their characteristics.

MNPs, M_1_M_2_NPs	Precursor	Stabilizer	Type plasma U, V	Max. abs. peak (*λ*_max_) (nm)	Particle shape and size (nm)	Ref.
AgNPs	AgNO_3_	SC	30 kV, 9.1 kHz	369–416	5.4–17.8	[14]
	AgNO_3_, EtOH	—	6000	403, 412, 420	8–10	[15]
	AgNO_3_	PVA	1500–2500	∼410	10 ± 7	[16]
	AgNO_3_	—	50 kHz and 2.5 *μ*s, 3500 (max)	∼400–410	Spherical, ∼10	[17]
	Ag sacrificial electrode	PVP	175–275	394–417	5–10	[18]
	AgNO_3_	PEC, SDS	1100	409.4, 409.8	9.33 ± 3.37 PEC-AgNPs 28.3 ± 11.7 SDS-AgNP	[19]
	Ag sacrificial electrode	—	Bipolar pulses 3.8 kV, 5 kHz	410.03–415.39	25–350	[20]

AuNPs	Au sacrificial electrode	Without stabilizer	Plasma sputtering, 20 kHz	511	Spherical, ∼3.5	[21]
	H[AuCl_4_]	Lysine	Pulsed discharge plasma	510–550	<20	[22]
	H[AuCl_4_]	Without stabilizer	From ∼2000 to ∼800	From 532 to 581 (from 2.5 *μ*M to 1 mM HAuCl_4_)	5–200	[23]
	H[AuCl_4_]	Without stabilizer	5000	552 ± 1; 532 ± 1	3.2 ± 0.4; 0.8 ± 0.5	[24]
	H[AuCl_4_]	GEL, PVP, PVA	1100–1300	531, 534, 535	27, 73, 92	[25]
	H[AuCl_4_]	SDS	1600, 2400, 3200	—	150 NPs (1 nm NCs)	[26]
	H[AuCl_4_]	SC	6800, 90 kHz	584, 566, 535	18.2 ± 9.0, 32.9 ± 14.1, 180.6 ± 20.5	[27]
	H[AuCl_4_]	Fructose	2000 to ignite the microplasma	∼530	∼33 (25°C), 37 (70°C)	[28]

PtNPs	Pt electrode	—	Low-voltage, low-frequency technique: 440, 500–100 Hz	—	≤10	[29]
PtNPs	H_2_[PtCl_6_]	Dextran and without stabilizer	15000 peak-to-peak with a frequency of 25 kHz	−	3–5	[30]
PdNPs	PdCl_2_				3–15	
RhNPs	RhCl_3_				4.7 ± 1	
CuNPs	CuCl_2_	GEL	900, 20 kHz frequency	∼580	Spherical (33.7 ± 5.8), cubic (19.2 ± 3.3), and hexagonal (20.3 ± 2.9)	[31]
NiNPs	Ni(NO_3_)_2_	—	70	362 and 380	Spherical, ∼15	[32]
	NiCl_2_	CTAB, SDS	250, 25–30 kHz	—	20–100	[33]
ZnNPs	Zn sacrificial electrode	Without stabilizer	70	—	13.97–22.64	[34]
MnNPs	MnCl_2_	CTAB	Pulsed discharge, 250.10, 30 kHz	—	5–10, 20–50	[35]
(PtM)NPs (*M* = cu, ag, pd)	Sucrifical electrodes	—	Pulsed plasma discharge, 1000, 20 kHz	—	4–6	[36]
(PtAg) NPs	Sucrifical Pt and Ag electrodes	—	1000, 30 kHz. pulse duration from 1.3 to 2.3 ms	—	<5	[37]
(AgPt)NPs	Sucrifical Ag and Pt electrodes	SDS	Unipolar pulsed dc to electrodes, 500, 3 *μ*s, 15 kHz	406.28–414.63	∼5	[38]
(PtPd)NPs	Sucrifical Pt and Pd electrodes	—	700, pulse width and frequency were 2 *μ*s and 20 kHz	—	2–3	[39]
(PtAu)NPs	Sucrifical Pt and Au electrodes	PEG	800 (breakdown voltage), pulsed DC 10–20 kHz (width 1–2 ls)	—	1.5 ± 1.0	[40]
(AuPd)NPs	H[AuCl_4_] and H_2_[PdCl_4_]	TCI	1500 W	—	∼3	[41]
(NiCu)NPs	Ni(NO_3_)_2_ and Cu(NO_3_)_2_	CTAB		—	Spherical, 50–200	[42]
(CoNi)NPs	Sucrifical Co and Ni electrodes	—	7 kV, 10 Hz	—	>100	[43]
(NiCu)NPs	Sucrifical CuNi electrodes	—	160	—	<200	[44]
(NiCr)NPs	Sucrifical NiCr electrodes					

CTAB, cethyltrimethylammonium bromide; GEL, gelatin; PEC, pectins; PEG, polyethylene glycol; PVP, polyvinylpyrrolidone; PVA, polyvinyl alcohol; SC, sodium citrate; SDS, sodium dodecyl sulfate, CH_3_(CH_2_)_11_OSO_3_Na; TCI, *α*-thioglycerol.

**Table 2:** Antibacterial properties of colloidal solutions of silver nanoparticles, synthesized by microplasma discharge in 0.1 mmol·L^−1^ AgNO_3_ and stabilized with polyacrylate solutions.

Species of bacteria	Exposure time (h)	Quantity (CFU/cm^3^)	Bactericidal action
*S. aureus* ATCC 25923 (F-49)	1	120	–
	6	50	–
	18	50	–
	48	30	–

*E. coli* ATCC 25922 (F-50)	1	70	–
	6	Not found	+
	18	Not found	+
	48	Not found	+

CFU, colony-forming units; +, pronounced antimicrobial (disinfecting) effect (no growth of microorganisms); –, no antimicrobial (disinfectant) action (available growth of microorganisms).

**Table 3:** Antibacterial properties of colloidal solutions of silver nanoparticles, synthesized by microplasma discharge in 0.2 mmol·L^−1^ AgNO_3_ and stabilized with polyacrylate solutions.

Species of bacteria	Exposure time (h)	Quantity (CFU/cm^3^)	Bactericidal action
*S. aureus* ATCC 25923 (F-49)	1	100	–
	6	50	–
	18	Not found	+
	48	Not found	+

*E. coli* ATCC 25922 (F-50)	1	40	–
	6	Not found	+
	18	Not found	+
	48	Not found	+

CFU, colony-forming units; +, pronounced antimicrobial (disinfecting) effect (no growth of microorganisms); –, no antimicrobial (disinfectant) action (available growth of microorganisms).

**Table 4:** Fungicidal properties of colloidal solutions of silver nanoparticles, synthesized by microplasma discharge in 0.1 mmol·L^−1^ AgNO_3_ and stabilized with polyacrylate solution.

Species of mushrooms	Exposure time (h)	Quantity (CFU/cm^3^)	Bactericidal action
*Candida* albicans ATCC 885–653	1	50	–
	6	9	–
	18	Not found	+
	48	Not found	+

**Table 5:** Fungicidal properties of colloidal solutions of silver nanoparticles, synthesized by microplasma discharge in 0.2 mmol·L^−1^ AgNO_3_ and stabilized with polyacrylate solution.

Species of mushrooms	Exposure time (h)	Quantity (CFU/cm^3^)	Bactericidal action
*Candida* albicans ATCC 885–653	1	40	–
	6	8	–
	18	Not found	+
	48	Not found	+

## Data Availability

The data used to support the findings of this study are included within the article.
